The article "A Deep Spiking Neural Network Anomaly Detection Method" was retracted in 2023. Reasons: signs of a paper mill; suspected computer-generated content; unreliable results or conclusions; concerns about the data.

# A Deep Spiking Neural Network Anomaly Detection Method

**DOI:** 10.1155/2022/6391750

**Published:** 2022-09-21

**Authors:** Lixia Hu, Ya Liu, Wei Qiu

**Affiliations:** ^1^Department of Computer Science and Engineering, Langfang Polytechnic Institute, Langfang 065000, China; ^2^Department of Electrical Automation, Hebei University of Water Resources and Electric Engineering, Cangzhou 061001, China

## Abstract

Cyber-attacks on specialized industrial control systems are increasing in frequency and sophistication, which means stronger countermeasures need to be implemented, requiring the designers of the equipment in question to re-evaluate and redefine their methods for actively protecting against advanced mass cyber-attacks. The attacks in question have huge motivations, ranging from corporate espionage to political targets, but in any case, they have a substantial financial impact and severe real-world implications. It should also be said that it is challenging to defend against cyber threats because a single point of entry can be enough to destroy an entire organization or put it out of business. This paper examines threats to the digital security of vibration monitoring systems used in petroleum infrastructure protection services, such as pipelines, pumps, and tank farms, where malicious interventions can cause explosions, fires, or toxic releases, with incalculable economic and environmental consequences. Specifically, a deep spiking neural network anomaly detection method is presented, which models the spike sequences and the internal presentation mechanisms of the information to discover with very high accuracy anomalies in vibration analysis systems used in oil infrastructure protection services. This is achieved by simulating the complex structures of the human brain and the way neural information is processed and transmitted. This work uses a particularly innovative form of the Galves–Löcherbach Spiking Model (GLSM) [1], which is a spiking neural network model with intrinsic stochasticity, ideal for modeling complex spatiotemporal situations, which is enhanced with possibilities of exploiting confidence intervals by modeling optimally stochastic variable-length memory chains that have a finite state space.

## 1. Introduction

The advent of the 4th industrial revolution and the Internet of Things, communication between humans and machines is becoming more evident and functional [1]. The placement of sensors and smart applications and data extraction from the devices during their operation offer more and more accurate data to manage the process and control of the machines adequately. A big problem for industries is the shutdown of their infrastructure, which will cause significant economic damage [2]. The worst-case scenario is lured into unmanageable damaging scenarios, such as leaks and explosions, that can endanger thousands of people's lives or cause enormous ecological disasters. To avoid similar problems, industries add advanced techniques for monitoring the state of their infrastructures, vibration analysis, for example, is a procedure that monitors the operational status of active industrial equipment using data analytic methods [3, 4].

Specifically, vibration analysis is a method that analyzes the amount and frequency of machine vibrations and then utilizes this information to assess the machine's condition. Although the inner workings and formulae required to compute various vibrations may be sophisticated, all functions begin with high-speed laser sensors to capture and quantify them appropriately. Every time the machine operates, vibrations are generated. Laser sensors connected to the device produce a signal corresponding to the amount and frequency of the vibrations generated. All acquired data are sent immediately to the data collector, which records specific characteristics that can be used to determine infrastructure capacity [5].

Specifically, by attempting a technical evaluation of the characteristics of vibration analysis in industrial equipment, working conditions, and the features of vibrating elements, three main fields of interest are identified that can be exploited to extract useful information, namely:

1. Time Domain: the physical amount of vibration received by the laser sensors is converted into an electrical signal in the time domain and appears as a waveform.
2. Frequency Domain: by performing analysis on the waveforms, using frequencies versus amplitude, that is, spectrum analysis, we get the most thorough analysis of machine vibration.
3. Joint Domain: when the vibration signals change over time, it is helpful to compute more than one spectrum simultaneously. This is done using the standard time approach, Gabor-Wigner-Wavelet, which calcifies variants of the fast Fourier transform, including the short-time Fourier transform.

This procedure is a classical signal processing method that can condense measurements to extract information about some distant state of nature. From this point of view, signal processing can be described from different perspectives. To an acoustician, it is a tool to turn measured signals into useful information. To a sonar designer, it is one part of a sonar system. To an electrical engineer, it is often restricted to digitization, sampling, filtering, and spectral estimation. Mechanics and vibration process analyze these data to determine the machine's operating condition and identify potentially dangerous problems such as looseness, imbalance, misalignment, and lubrication issues. Unbalance, misfires, mechanical looseness, misalignment, tuning, motor faults, bent shafts, bearing failures, voids or bubbles in pumps, and critical speeds or environmental conditions, in particular, may be detected via vibration analysis [6].

One of the critical digital security tools of petroleum infrastructure, which extends and enhances vibration analysis systems, is anomaly detection systems. These systems are called upon to solve the complicated problem of identifying vibrations from abnormal events. As can be seen, these systems should be able to understand the underlying distribution of the data and single out outliers, which may be very few compared to the whole, but are of great importance.

So, the ability to formally express the dependencies between given multivariate events and to reason about the different states of the system over time is of great importance in the anomaly systems in question. This lies in the fact that infrequent events can provide precise expressions of patterns that can inform the system's future behavior and facilitate its more general supervision. As a result, it is critical to implement an event correlation system, which will also provide a common framework for representing the internal dynamics of a time series of events, especially the events associated with failure time data [7].

Standard probabilistic logics and corresponding tools provide reasoning over uncertain data, allowing the annotation of crucial facts with a probability value and using rules. However, in most cases, this is insufficient to express temporal correlations between observed patterns. To represent uncertain data and time dependencies, probabilistic temporal logic programming paradigms have been proposed in the literature, which is simple enough to model special situations. In contrast, improved precision data analysis technologies, such as neural network techniques, can use complex data such as vibration analysis data to extract a pattern or predict a future trend. These analyses are difficult to perform due to human observation and experience complexity [8]. The most important, perhaps, a disadvantage of simple artificial neural networks is the weakness they present in understanding their operation and the fact that the use of the mathematical relationships they implement does not necessarily guarantee that the neural network works efficiently, particularly in complicated circumstances where the time domain plays a vital role. This is because simple neural networks learn and train through a series of examples that are input as templates, automatically making the process of adequately selecting input data significantly train the neural network. For example, a severe simplifying assumption of simple neural networks concerns the view that the neural code used to exchange information between neurons is based on the average value of emitted spikes, a fact modeled as the propagation of continuous variables from one computing unit to another. But, it has been shown experimentally that not only is there not a constant propagation of spikes from which it is tentative to obtain their average value but also that the spikes appear periodically after the application of action and that the exact time of the spikes plays a significant role, if not the more critical role in neural information processing [9].

Spiking neural networks, on the other hand, allow for the thorough analysis and modeling of temporally determined information, utilizing important information such as neuronal firing rate, the relationship between a stimulus and individual or aggregate neural responses, the association between neuronal electrical activity as a whole them, and also the processes of polarization or depolarization of neuronal activity. These characteristics carry all the necessary elements for transmitting, analyzing, and utilizing information to the maximum extent. Such approaches extend the syntax and semantics of probabilistic logic programs, allowing reasoning about probabilities of points over time intervals using probabilistic time rules [10].

A complex spiking neural architecture is employed in this study to cover and avoid the simplifying assumptions and extensions of current essential neural network technologies. Specifically, a deep spiking neural network anomaly detection method is presented, which models the spike sequences and internal presentation mechanisms of the information to detect anomalies in vibration analysis systems used in oil infrastructure protection services with very high accuracy by simulating most realistically the complex structures of the human brain and the way neural information is processed and transmitted. In particular, a specialized GLSM is presented, which is ideal for modeling complex spatiotemporal situations, enhanced with confidence interval capabilities.

## 2. State-of-the-art

Recently, many studies have used spiking neural networks [11] in practical applications [12], the results of which show promise in the solution of real complex problems. Significant progress with their use has been made in areas such as speech recognition, machine vision, computer system security, complex learning systems from heterogeneous agents, and mechanisms that utilize associative memory and robotics.

In their study, Bariah et al. [1] utilized the characteristics of the Spiking Neural Network to construct an appropriate detector, address the problem of acquiring complicated features, collecting actionable data, and discriminating normal from differential expression. Throughout their training, they developed possible neurons, which spiked once they identified an abnormal pattern in the data. Their method was composed of three steps: implementing the weight values with the rank order method, expressing the real input data as peak values with Gaussian Receptive Fields, and finding the firing nodes that indicated anomalous data. They extended their method to anomalous data extracted from time series datasets. The experimental findings demonstrated that the proposed method could detect anomalies in information with an acceptable Classification Error Rate.

Demertzis et al. [11] published in 2017 an enhanced Spiking One-Class Anomaly Detection Framework relying on the developing Spiking Neural Network technique, which enabled a novel implementation of the one-class supervised classification. Because it is trained solely with data describing the usual function of an Industrial Control System, it is able to identify deviating trends and anomalies related to Advanced Persistent Threat campaigns. They logically structured information in a spatiotemporal fashion while simulating the activity of organic brain cells in the most practical style. Length and intensity of time bursts between neurons are essential parameters in the transmission of generated signals. In addition, they incorporated AI technology at the level of real-time evaluation of industrial machinery, which significantly strengthens the protective mechanisms of vital infrastructures, managing the interrelations of ICS at all times and making it much simpler to detect APT attempts, as they discovered.

Stratton et al. [13] examined Spiking Neural Networks by employing text stream anomaly detection. They demonstrated that SNNs are well-suited for recognizing unusual strings, that they might learn quickly, and that numerous SNN architectural and learning modifications can increase anomaly detection efficiency. Anomaly detection must be automated in order to manage big quantities of information and meet real-time processing restrictions. Spiking Neural Networks offer the ability to perform well with AD, particularly for edge applications where it must be limited, easily adaptive, independent, and dependable. Upcoming research will employ more comprehensive and difficult training datasets and directly compare the performance of SNNs and Deep Neural Networks educated on a same dataset using systems of comparable size.

Utilizing spiking neural networks, Dennler et al. [10] suggested a neuromorphic method for dynamic analysis that may be used to a variety of circumstances. Vibration patterns provide vital data on health condition of operating equipment, which is typically utilized in preventative maintenance duties for big manufacturing systems. Nonetheless, the scale, sophistication, and power budget needed by conventional ways to exploit this information are often too expensive for various applications such as selfdriving automobiles, uncrewed aerial vehicles, and automation. They created a spike-based end-to-end system that works unsupervised online to identify system abnormalities using vibration data, leveraging building blocks compatible with analog-digital artificial neural circuits. They proved that the suggested approach met or surpassed state-of-the-art performance on two publicly available datasets. In addition, they implemented a proof-of-concept on an asynchronous artificial neural processor device, advancing the development and operation of independent reduced end devices for continuous vibration analysis.

Maciag et al. [14] found anomalies in stream data without supervision as the primary study subject in their research work. Specifically, they proposed an Online Growing Spiking Neural Network for Unsupervised Anomaly Detection method. Unlike the Online Growing Spiking Neural Network, it worked unsupervised and did not partition output neurons into discrete judgment classes. However, collecting adequate instruction data with labeled irregularities for labeled data of an automated tracking that may subsequently be implemented to spot actual abnormalities in data in real-time is challenging in many cases. As a result, it is critical to building anomaly detectors that can identify abnormalities even in the absence of labeled training data. To identify abnormalities, they used a two-step technique. The proposed detector outperforms existing methods published in the literature for data streams in experimental comparisons with state-of-the-art unassisted and semisupervised sensors of deviations in datasets from known dataset repositories.

Using an adjusted evolving Spiking Neural Network, Dennis et al. [9] presented a model for detecting anomalies in flowing multivariate time series. They contributed a substitute rank-order-based autoencoder that used the precise times of incoming spikes for adjusting network parameters, an adapted, real-time-capable, and reliable learning algorithm for multivariate data based on multidimensional Gaussian Receptive Fields, and a constant outlier scoring function for enhanced interpretability of the classifications. The potential applications for this type of algorithm are diverse. It extends from tracking digital machinery and preventative maintenance to big data healthcare datalogger analysis applications. Spiking algorithms are particularly effective in time-dependent information processing. They showed the prototype's effectiveness on a synthetic dataset based on a reference point containing various types of anomalies, comparing it to other streaming anomaly detection methodologies and demonstrating that their algorithm performed better at detecting anomalies while requiring fewer computational resources for processing high-dimensional data.

## 3. Vibration Analysis Data

Failures related to bearings and lubrication systems are one of the leading causes of forced outages in turbine systems [15]. In some cases, machinery can explode, causing extensive damage to other equipment and even human casualties. Transverse vibrations in high-speed shafts, mainly in turbine engines, can capture the coexistence of transverse cracking and wear in bearings under certain conditions. A shaft is considered a high-speed shaft if it rotates at a speed greater than the critical speed, that is, a speed at which transverse vibrations of significant magnitude occur. This analysis focuses on motion oscillation problems in the critical and postcritical speed ranges, determining the frequency ranges for natural vibrations and critical speeds, and evaluating stability, specifically, stability within the case-specific critical range [16].

In particular, the analysis considers the case of the rotor bearing system using boundary conditions that combine the rotor shear force and the fluid frame (flange) forces at the points where the bearings contact. The behavior of the bearing is assumed to be nonlinear since its dynamic properties are captured by the actual function of its periodic position and linear velocity at a given time. It should be noted that material damping is introduced into the rotor model to achieve time-domain solutions, even at critical speeds, independent of the length of time the system is in resonance. In such cases, the analysis gives response results too close to or even higher than the radial distance and is considered insufficient. The model has an initial condition with time-dependent boundary values. This is obtained by expressing flange forces as a function of rotor force shear [17].

The initial depiction of the operating conditions at random times is shown diagrammatically in Figure 1.

The main objective of the current work is to investigate the system's dynamics with characteristics in both the frequency and time domains under the assumption of a continuous rotor in nonlinear conditions of bearing operations [18].

The approach looks for elements such as rotor motion, rotational inertia, punching deformation, and torque due to power transmission, considering the gyroscopic effect. Specifically, the function that is considered for the vertical movement is [19]:

(1) $$\begin{array}{c} E^{*}I_{j}\frac{\partial^{4}Y_{j}}{\partial x^{4}}-\frac{E^{*}I_{j}\rho }{kG^{*}}\frac{\partial^{4}Y_{j}}{\partial x^{2}\partial t^{2}}+T\frac{\partial^{3}Z_{j}}{\partial x^{3}}-\frac{T\rho }{kG^{*}}\frac{\partial^{3}Z_{j}}{\partial x\partial t^{2}}+\rho A_{j}\frac{\partial^{2}Y_{j}}{\partial t^{2}}\\ -\rho A_{j}r_{0}^{2}\left[\left(\frac{\partial^{4}Y_{j}}{\partial x^{2}\partial t^{2}}-\frac{\rho }{kG^{*}}\frac{\partial^{4}Y_{j}}{\partial t^{4}}\right)+2\Omega \left(\frac{\partial^{3}Z_{j}}{\partial x^{2}\partial t}-\frac{\rho }{kG^{*}}\frac{\partial^{3}Z_{j}}{\partial t^{3}}\right)\right]=0\cdot \end{array}$$

While for the horizontal movement, it is the:

(2) $$\begin{array}{c} E^{*}I_{j}\frac{\partial^{4}Z_{j}}{\partial x^{4}}-\frac{E^{*}I_{j}\rho }{kG^{*}}\frac{\partial^{4}Z_{j}}{\partial x^{2}\partial t^{2}}-T\frac{\partial^{3}Y_{j}}{\partial x^{3}}+\frac{T\rho }{kG^{*}}\frac{\partial^{3}Y_{j}}{\partial x\partial t^{2}}+\rho A_{j}\frac{\partial^{2}Z_{j}}{\partial t^{2}}\\ -\rho A_{j}r_{0_{j}}^{2}\left[\left(\frac{\partial^{4}Z_{j}}{\partial x^{2}\partial t^{2}}-\frac{\rho }{kG^{*}}\frac{\partial^{4}Z_{j}}{\partial t^{4}}\right)-2\Omega \left(\frac{\partial^{3}Y_{j}}{\partial x^{2}\partial t}-\frac{\rho }{kG^{*}}\frac{\partial^{3}Y_{j}}{\partial t^{3}}\right)\right]=0\cdot \end{array}$$

Given the:

Complex Young modulus:

(3) $$\begin{array}{c} E^{*}=E\left(1+i\cdot \eta \right)\cdot \end{array}$$

Complex shear modulus:

(4) $$\begin{array}{c} G^{*}=G\cdot \left(1+i\cdot \eta \right)\cdot \end{array}$$

The radius of gyration of each step:

(5) $$\begin{array}{c} r_{0_{j}}=\sqrt{\frac{I_{j}}{A_{j}}}\cdot \end{array}$$

Boundary conditions are constraints necessary to solve a boundary value problem. A boundary value problem is a differential equation (or system of differential equations) to be solved in a domain on whose boundary a set of conditions is known. Aside from the boundary condition, boundary value problems are also classified according to the type of differential operator involved. These categories are further subdivided into linear and various nonlinear types. For an elliptic operator, one discusses elliptic boundary value problems. For a hyperbolic operator, one discusses hyperbolic boundary value problems.

Many significant problems, such as flow driven by moving objects, free-surface flow, flow involving air bubbles, flow accompanying phase transition, and fluid-structure interaction, are moving boundary problems. In dealing with such boundaries with movement or deformation, the traditional mesh methods such as finite difference, finite element, and finite volume method generally encounter difficulties in accurately calculating the geometric form of the border.

Numerous numerical analyses have been performed to study problems with large interfacial deformation, such as free-surface and multiphase flows. However, besides the aforementioned valuable characteristics, the vibration calculation algorithm of the particle method also has a severe negative aspect: difficulty in the treatment of fixed boundaries (e.g., solid walls). In the mesh-free framework of calculation, spatial derivatives of the physical quantities (e.g., velocity and pressure) and the value of the particle number density are calculated by referencing the relative positions of surrounding particles that are present inside the practical domain. Still, the affective domain is truncated by the actual boundary for particles near the real boundary.

In our approach, boundary conditions express the continuity and discontinuity of shear force, bending moment, pitch, and displacement of the rotor depending on where the boundary exists. Specifically, the following boundary conditions are expressed in equations:

Slope:

(6) $$\begin{array}{c} S_{Y_{j,R}}\left(x,t\right)=\frac{\partial }{\partial x}\left(Y_{j,R}\left(x,t\right)\right),S_{Y_{J,I}}\left(x,t\right)=\frac{\partial }{\partial x}\left(Y_{j,I}\left(x,t\right)\right)\text{,}\\ S_{Z_{J,R}}\left(x,t\right)=\frac{\partial }{\partial x}\left(Z_{j,R}\left(x,t\right)\right),S_{Z_{J,I}}\left(x,t\right)=\frac{\partial }{\partial x}\left(Z_{j,I}\left(x,t\right)\right)\cdot \end{array}$$

Bending moment:

(7) $$\begin{array}{c} M_{Y_{J,R}}\left(x,t\right)=EI_{j}\frac{\partial^{2}}{\partial x^{2}}\left(Y_{j,R}\left(x,t\right)\right)-EI_{j}\eta \frac{\partial^{2}}{\partial x^{2}}\left(Y_{j,I}\left(x,t\right)\right)\text{,}\\ M_{Y_{J,I}}\left(x,t\right)=EI_{j}\frac{\partial^{2}}{\partial x^{2}}\left(Y_{j,I}\left(x,t\right)\right)+EI_{j}\eta \frac{\partial^{2}}{\partial x^{2}}\left(Y_{j,R}\left(x,t\right)\right)\text{,}\\ M_{Z_{J,R}}\left(x,t\right)=EI_{j}\frac{\partial^{2}}{\partial x^{2}}\left(Z_{j,R}\left(x,t\right)\right)-EI_{j}\eta \frac{\partial^{2}}{\partial x^{2}}\left(Z_{j,I}\left(x,t\right)\right)\text{,}\\ M_{Z_{J,I}}\left(x,t\right)=EI_{j}\frac{\partial^{2}}{\partial x^{2}}\left(Z_{j,I}\left(x,t\right)\right)+EI_{j}\eta \frac{\partial^{2}}{\partial x^{2}}\left(Z_{j,R}\left(x,t\right)\right)\cdot \end{array}$$

Shearing force:

(8) $$\begin{array}{c} V_{Y_{J,R}}\left(x,t\right)=EI_{j}\left(\frac{\partial^{3}Y_{j,R}\left(x,t\right)}{\partial x^{3}}-\eta \frac{\partial^{3}Y_{j,I}\left(x,t\right)}{\partial x^{3}}\right)-\rho A_{j}r_{0,j}^{2}\left(G_{1,R}\left(x,t\right)+2\Omega G_{2,R}\left(x,t\right)\right)\text{,}\\ V_{Y_{J,t}}\left(x,t\right)=EI_{j}\left(\eta \frac{\partial^{3}Y_{j,R}\left(x,t\right)}{\partial x^{3}}+\frac{\partial^{3}Y_{j,I}\left(x,t\right)}{\partial x^{3}}\right)-\rho A_{j}r_{0j}^{2}\left(G_{1_{j,t}}\left(x,t\right)+2\Omega G_{2,t}\left(x,t\right)\right)\text{,}\\ V_{Z_{J,R}}\left(x,t\right)=EI_{j}\left(\frac{\partial^{3}Z_{j,R}\left(x,t\right)}{\partial x^{3}}-\eta \frac{\partial^{3}Z_{j,I}\left(x,t\right)}{\partial x^{3}}\right)-\rho A_{j}r_{0j}^{2}\left(G_{3_{j,R}}\left(x,t\right)+2\Omega G_{4_{4,R}}\left(x,t\right)\right)\text{,}\\ V_{Z_{J,l}}\left(x,t\right)=EI_{j}\left(\eta \frac{\partial^{3}Z_{j,R}\left(x,t\right)}{\partial x^{3}}+\frac{\partial^{3}Z_{j,I}\left(x,t\right)}{\partial x^{3}}\right)-\rho A_{j}r_{0j}^{2}\left(G_{3_{j,l}}\left(x,t\right)+2\Omega G_{4_{,n}}\left(x,t\right)\right)\cdot \end{array}$$

Using finite frontal differences of the first order in the time domain, the terms are expressed as shown in the following equations:

Real vertical slope:

(9) $$\begin{array}{c} G_{1_{j,R}}\left(x,t\right)=\frac{S_{Y_{j,R}}\left(x,t\right)-2S_{Y_{j,R}}\left(x,t-\Delta t\right)+S_{Y_{j,R}}\left(x,t-2\Delta t\right)}{\Delta t^{2}}\cdot \end{array}$$

Imaginary vertical slope:

(10) $$\begin{array}{c} G_{1_{j,t}}\left(x,t\right)=\frac{S_{Y_{j,t}}\left(x,t\right)-2S_{Y_{j,t}}\left(x,t-\Delta t\right)+S_{Y_{j,t}}\left(x,t-2\Delta t\right)}{\Delta t^{2}}\cdot \end{array}$$

Real vertical slope velocity:

(11) $$\begin{array}{c} G_{2_{j,R}}\left(x,t\right)=\frac{S_{Y_{j,R}}\left(x,t\right)-S_{Y_{j,R}}\left(x,t-\Delta t\right)}{\Delta t}\cdot \end{array}$$

Imaginary vertical slope velocity:

(12) $$\begin{array}{c} G_{2_{j,I}}\left(x,t\right)=\frac{S_{Y_{j,I}}\left(x,t\right)-S_{Y_{j,I}}\left(x,t-\Delta t\right)}{\Delta t}\cdot \end{array}$$

Real horizontal slope:

(13) $$\begin{array}{c} G_{3_{j,R}}\left(x,t\right)=\frac{S_{Z_{j,R}}\left(x,t\right)-2S_{Z_{j,R}}\left(x,t-\Delta t\right)+S_{Z_{j,R}}\left(x,t-2\Delta t\right)}{\Delta t^{2}}\cdot \end{array}$$

Imaginary horizontal slope:

(14) $$\begin{array}{c} G_{3_{j,t}}\left(x,t\right)=\frac{S_{Z_{j,t}}\left(x,t\right)-2S_{Z_{j,t}}\left(x,t-\Delta t\right)+S_{Z_{j,t}}\left(x,t-2\Delta t\right)}{\Delta t^{2}}\cdot \end{array}$$

Real horizontal slope velocity:

(15) $$\begin{array}{c} G_{4_{j,R}}\left(x,t\right)=\frac{S_{Z_{j,R}}\left(x,t\right)-S_{Z_{j,R}}\left(x,t-\Delta t\right)}{\Delta t}\cdot \end{array}$$

Imaginary horizontal slope velocity:

(16) $$\begin{array}{c} G_{4_{j,I}}\left(x,t\right)=\frac{S_{Z_{j,I}}\left(x,t\right)-S_{Z_{j,I}}\left(x,t-\Delta t\right)}{\Delta t}\cdot \end{array}$$

Real vertical acceleration:

(17) $$\begin{array}{c} G_{5_{j,R}}\left(x,t\right)=\frac{Y_{j,R}\left(x,t\right)-2Y_{j,R}\left(x,t-\Delta t\right)+Y_{j,R}\left(x,t-2\Delta t\right)}{\Delta t^{2}}\cdot \end{array}$$

Imaginary vertical acceleration:

(18) $$\begin{array}{c} G_{5_{j,I}}\left(x,t\right)=\frac{Y_{j,I}\left(x,t\right)-2Y_{j,I}\left(x,t-\Delta t\right)+Y_{j,I}\left(x,t-2\Delta t\right)}{\Delta t^{2}}\cdot \end{array}$$

Real horizontal acceleration:

(19) $$\begin{array}{c} G_{6_{j,R}}\left(x,t\right)=\frac{Z_{j,R}\left(x,t\right)-2Z_{j,R}\left(x,t-\Delta t\right)+Z_{j,R}\left(x,t-2\Delta t\right)}{\Delta t^{2}}\cdot \end{array}$$

Imaginary horizontal acceleration:

(20) $$\begin{array}{c} G_{6_{j,l}}\left(x,t\right)=\frac{Z_{j,I}\left(x,t\right)-2Z_{j,I}\left(x,t-\Delta t\right)+Z_{j,I}\left(x,t-2\Delta t\right)}{\Delta t^{2}}\cdot \end{array}$$

Real boundary conditions.

Vertical plane bearings:

(21) $$\begin{array}{c} \sigma_{1}=M_{Y_{1,R}}\left(0,t\right)\text{,}\\ \sigma_{2}=M_{Y_{2,R}}\left(L,t\right)\text{,}\\ \sigma_{3}=F_{Y_{1,R}}-{\left.EI_{1}\frac{\partial^{3}Y_{ST_{1}}}{\partial x^{3}}\right|}_{x=0}-V_{Y_{1,R}}\left(0,t\right)\text{,}\\ \sigma_{4}=F_{Y_{2,R}}+{\left.EI_{2}\frac{\partial^{3}Y_{ST_{2}}}{\partial x^{3}}\right|}_{x=L}+M_{Y_{2,R}}\left(L,t\right)\cdot \end{array}$$

Location of floor:

(22) $$\begin{array}{c} \sigma_{5}=M_{Y_{2,R}}\left(L_{1},t\right)-M_{Y_{1,R}}\left(L_{1},t\right)\text{,}\\ \sigma_{6}=M_{Y_{2,R}}\left(L_{1},t\right)-M_{Y_{1,R}}\left(L_{1},t\right)+I_{P}\Omega G_{2_{2,R}}\left(L_{1},t\right)+I_{T}G_{3_{2,R}}\left(L_{1},t\right)\text{,}\\ \sigma_{7}=V_{Y_{2,R}}\left(L_{1},t\right)-V_{Y_{1,R}}\left(L_{1},t\right)-F_{u_{Y}}+E_{F}+m_{d}G_{5_{2,R}}\left(L_{1},t\right)\text{,}\\ \sigma_{8}=Y_{2,R}\left(L_{1},t\right)-Y_{1,R}\left(L_{1},t\right)\cdot \end{array}$$

Horizontal plane bearings:

(23) $$\begin{array}{c} \sigma_{9}=M_{Z_{1,R}}\left(0,t\right)\text{,}\\ \sigma_{10}=M_{Z_{2,R}}\left(L,t\right)\text{,}\\ \sigma_{11}=F_{Z_{1,R}}-V_{Z_{1,R}}\left(0,t\right)\text{,}\\ \sigma_{12}=F_{Y_{2,R}}+V_{Z_{2,R}}\left(L,t\right)\cdot \end{array}$$

Location of floor:

(24) $$\begin{array}{c} \sigma_{13}=S_{Z_{2,R}}\left(L_{1},t\right)-S_{Z_{1,R}}\left(L_{1},t\right)\text{,}\\ \sigma_{14}=M_{Z_{2,R}}\left(L_{1},t\right)-M_{Z_{1,R}}\left(L_{1},t\right)+I_{P}\Omega G_{4_{2,R}}\left(L_{1},t\right)-I_{T}G_{1_{2,R}}\left(L_{1},t\right)\text{,}\\ \sigma_{15}=V_{Z_{2,R}}\left(L_{1},t\right)-V_{Z_{1,R}}\left(L_{1},t\right)-F_{u_{Z}}+m_{d}G_{6_{2,R}}\left(L_{1},t\right)\text{,}\\ \sigma_{16}=Z_{2,R}\left(L_{1},t\right)-Z_{1,R}\left(L_{1},t\right)\cdot \end{array}$$

Imaginary boundary conditions.

Vertical plane bearings:

(25) $$\begin{array}{c} \sigma_{17}=M_{Y_{1,t}}\left(0,t\right)\text{,}\\ \sigma_{18}=M_{Y_{2,t}}\left(L,t\right)\text{,}\\ \sigma_{19}=F_{Y_{,,}}-{\left.EI_{1}\frac{\partial^{3}Y_{ST_{1}}}{\partial x^{3}}\right|}_{x=0}-V_{Y_{1,t}}\left(0,t\right)\text{,}\\ \sigma_{20}=F_{Y_{2,I}}+{\left.EI_{2}\frac{\partial^{3}Y_{ST_{2}}}{\partial x^{3}}\right|}_{x=L}+V_{Y_{2,I}}\left(L,t\right)\cdot \end{array}$$

Location of floor:

(26) $$\begin{array}{c} \sigma_{21}=S_{Y_{2,t}}\left(L_{1},t\right)-S_{Y_{1,t}}\left(L_{1},t\right)\text{,}\\ \sigma_{22}=M_{Y_{2,i}}\left(L_{1},t\right)-M_{Y_{1,t}}\left(L_{1},t\right)+I_{P}\Omega G_{2_{2,t}}\left(L_{1},t\right)+I_{T}G_{3_{2,t}}\left(L_{1},t\right)\text{,}\\ \sigma_{23}=V_{Y_{2,i}}\left(L_{1},t\right)-V_{Y_{1,t}}\left(L_{1},t\right)-F_{u_{Y}}+E_{F}+m_{d}G_{S_{2,i}}\left(L_{1},t\right)\text{,}\\ \sigma_{24}=Y_{2,I}\left(L_{1},t\right)-Y_{1,I}\left(L_{1},t\right)\cdot \end{array}$$

Horizontal plane bearings:

(27) $$\begin{array}{c} \sigma_{25}=M_{Z_{1,I}}\left(0,t\right)\text{,}\\ \sigma_{26}=M_{Z_{2,I}}\left(L,t\right)\text{,}\\ \sigma_{27}=F_{Z_{1,I}}-V_{Z_{1,I}}\left(0,t\right)\text{,}\\ \sigma_{28}=F_{Y_{2,I}}+V_{Z_{2,I}}\left(L,t\right)\cdot \end{array}$$

Location of floor:

(28) $$\begin{array}{c} \sigma_{29}=S_{Z_{2,I}}\left(L_{1},t\right)-S_{Z_{1,I}}\left(L_{1},t\right)\text{,}\\ \sigma_{30}=M_{Z_{2,I}}\left(L_{1},t\right)-M_{Z_{1,I}}\left(L_{1},t\right)+I_{P}\Omega G_{4_{2,I}}\left(L_{1},t\right)-I_{T}G_{1_{2,I}}\left(L_{1},t\right)\text{,}\\ \sigma_{31}=V_{Z_{2,I}}\left(L_{1},t\right)-V_{Z_{1,I}}\left(L_{1},t\right)-F_{u_{Z}}+m_{d}G_{6_{2,I}}\left(L_{1},t\right)\text{,}\\ \sigma_{32}=Z_{2,I}\left(L_{1},t\right)-Z_{1,I}\left(L_{1},t\right)\cdot \end{array}$$

Before extracting features, the recorded signals received appropriate preprocessing, intending to suppress unwanted distortions and enhance the most critical features for further processing [20]. Specifically, first, the signals were filtered using a digital bandpass filter of order 5 with a range of 0.5-30 Hz. We use low frequencies because the parts of the signals that contain essential information may be in lower frequency bands. Also, since the effect of filtering on the signals is weighted, that is, greater in the center of the filter values, not all the interference of the 50 Hz band is neutralized. As a result, bandpass filtering must be applied to the signals immediately after bandpass filtering. A band-stop filter with a narrow rejection band and a high-quality factor *Q* = 30 is used to attenuate frequencies near 50 Hz. Accordingly, after filtering, we proceed to normalize the signals. For each trial and electrode, the average of the signal is subtracted from each time sample. The result of the previous operation is divided by the standard deviation, as shown by the following equation:

(29) $$\begin{array}{c} x_{i}^{*}\left(t\right)=\frac{x_{i}\left(t\right)-{\bar{x}}_{i}}{SD{\left(x\right)}_{i}}\cdot \end{array}$$

To calculate the band power characteristics for each of the three channels containing useful information C3, C4, and CZ, the parts of the signal corresponding to the quiescent state are trimmed based on the quiescent times. On the resulting signals after clipping, we apply bandpass filtering to 72 frequency bands using different overlapping narrow bands between 8 Hz and 30 Hz. The characteristics are calculated by subtracting the power values of the resting parts from the power values of the parts corresponding to vibrations. Then, we apply bandpass filtering to the resting window using a digital filter of order 5 at 8-12 Hz and 13-25 Hz, since the power during the resting state serves as a reference point in both frequency bands. The segments are also filtered with the same filter at the frequencies 8-12 Hz and 13-30 Hz, respectively. We get the power samples from the parts of the original signal that have been cut and filtered by squaring the available amplitude samples. To calculate the final features, we subtract the average power of a trial during the windows from the filtered resting time intervals. Similarly, the mean of single-trial power samples during rest windows is subtracted from the band-filtered rest intervals [21].

Finally, for pattern estimation and feature distribution, it is approximated by the logarithm of the variance of a band-pass filtered signal at specific time intervals so that [22]:

(30) $$\begin{array}{c} u_{c}\left(i\right)=\frac{2}{\tau -1}\overset{k_{n}+\tau -1}{\underset{j=t_{n}}{\sum }}\;{\left(x_{y}-{\bar{x}}_{i}\right)}^{2}\cdot \end{array}$$

For each channel, the logarithmic band power characteristic is defined by the following formula:

(31) $$\begin{array}{c} BP_{c}\left(i\right)=\log\;\left(u_{e}\left(i\right)\right)\cdot \end{array}$$

Each class and each channel are calculated by taking the median of the average data variances for all trials. We use the median as it is more robust to extreme values. The total band power is written as follows:

(32) $$\begin{array}{c} {\tilde{BP}}_{c}^{X}=\log\;\left({\tilde{u}}_{e}\right)\cdot \end{array}$$

Thus, we can now define the Pattern Difference PDc for channels C3 and C4 between the two problem classes N (normal) and A (abnormal) [23]:

(33) $$\begin{array}{c} PD_{C3}={\tilde{BP}}_{C3}^{N}-{\tilde{BP}}_{C3}^{A}\text{,}\\ PD_{C4}={\tilde{BP}}_{C4}^{N}-{\tilde{BP}}_{C4}^{A}\cdot \end{array}$$

When PD pattern difference is calculated on small sub-bands of a dataset, the results show in which frequency bands the reduction in band power due to vibrations is most prominent. Since the specific band varies between subjects and recording sessions, results will vary accordingly along the band.

## 4. Proposed Deep Spiking Neural Architecture

The suggested application's primary goal is anomaly identification, which finds unusual occurrences, features, or observations that are unusual because they deviate considerably from typical patterns or behaviors. Anomalies in the data should be separated by an algorithmic system that can identify and appropriately classify standard deviations associated with marginal uses of the equipment relative to outliers, noise, novel uses, and exceptions. The modeling in question requires a neural architecture where the exchange of information between random neurons occurring at random synapses can create a specialized functional structure connecting neurons through random discrete events. Presynaptic and postsynaptic neurons can alternate their functions based on probabilistic functions. A neuron can simultaneously be presynaptic to some synapses and postsynaptic to others, depending on how it participates in them.

Based on the above requirements, a particularly innovative form of the Galves–Löcherbach Spiking Model (GLSM) [1] is used in this work, which is a spiking neural network model with inherent stochasticity, ideal for modeling complex spatiotemporal situations. A countable number of elements (idealized neurons) interact with sporadic near-instantaneous discrete events in the proposed GLSM (spikes or firings). Each neuron N fires independently at each moment, with a probability determined by the firing history of all neurons since the last time N fired. As a result, whenever a neuron fires, it forgets all initial spikes, including its own. This attribute represents the model's distinguishing trait. Specifically, we consider a stochastic chain (*X*_*t*_)_*t*∈*ℤ*_ that takes values in {0,1^*I*^} for some measurable set of neurons *I,* defined in a suitable probability space (Ω, *A*, *P*). For each neuron *i* at each time *t* ∈ *ℤ*, *X*_*t*_(*i*)=1, if neuron *i* is spiking at time *t* and *X*_*t*_(*i*)=0 otherwise. The global configuration of neurons at time *t* is denoted *X*_*t*_=(*X*_*t*_(*i*), *i* ∈ *I*). Filtering is defined as follows:

(34) $$\begin{array}{c} F_{t}=\sigma \left(X_{s},s\in Z,s\leq t\right),t\in Z\cdot \end{array}$$

For each neuron *i* ∈ *I*, for each instant *t* ∈ *Z* holds:

(35) $$\begin{array}{c} L_{t}^{i}=sup\left\{s<t:X_{s}\left(i\right)=1\right\}\cdot \end{array}$$

Which also translates as the last spike time of neuron *i* strictly before time *t*.

Then, we introduce a family of synaptic weights *W*_*j*⟶*i*_ ∈ *ℝ*, for *j* ≠ *i*, *W*_*j*⟶*j*_=0 for all *j*. *W*_*j*⟶*i*_ is the synaptic weight of neuron *j* to neuron *i*. We assume that the synaptic weights have the following uniform summation property [24]:

(36) $$\begin{array}{c} \underset{i\in I}{sup}\;\underset{j}{\sum }\;\left|W_{j⟶i}\right|<\infty \cdot \end{array}$$

At each time *t* (which is conditionally valid for the entire past), the domains are updated independently, which means that for any finite subset *J* ⊂ *I*, *a*_*i*_ ∈ {0,1}, *i* ∈ *J*, we have:

(37) $$\begin{array}{c} P\left(X_{t}\left(i\right)=a_{i},i\in J\;|\;F_{t-1}\right)=\prod_{i\in J}\;P\left(X_{t}\left(i\right)=a_{i}\;|\;F_{t-1}\right)\cdot \end{array}$$

Additionally, the probability of having a spike in neuron *i* at time *t* is given by the relation:

(38) $$\begin{array}{c} P\left(X_{t}\left(i\right)=1\;|\;F_{t-1}\right)=\phi_{i}\left(\underset{j}{\sum }\;W_{j⟶i}\overset{t-1}{\underset{s=L_{t}^{i}}{\sum }}\;g_{j}\left(t-s\right)X_{s}\left(j\right),t-L_{t}^{i}\right), \end{array}$$

where *ϕ*_*i*_ : *ℝ* × *ℕ*⟶[0,1] and *g*_*j*_ : *ℕ*⟶*ℝ*_+_ are measurable functions for all *i* ∈ *I*, *j* ∈ *I*. We assume that *ϕ*_*i*_ is uniformly continuous, that is, there exists a positive constant *γ* such that for all *s*, *s*′ ∈ *ℝ*, *n* ∈ *ℕ*, *i* ∈ *I* to be valid [25]:

(39) $$\begin{array}{c} \left|\phi_{i}\left(s,n\right)-\phi_{i}\left(s^{\prime },n\right)\right|\leq \gamma \left|s-s^{\prime }\right|\cdot \end{array}$$

The probability of a spike in the next time unit depends on the system's overall time evolution after the component's last spike time. We consider that the functions *ϕ*_*i*_ and *g*_*j*_ additionally satisfy the following assumptions and specifically there exists *δ* > 0 such that for all *i* ∈ *I*, *s* ∈ *R*, *n* ∈ *N* [26]:

(40) $$\begin{array}{c} \phi_{i}\left(s,n\right)\geq \delta \cdot \end{array}$$

So that:

(41) $$\begin{array}{c} G\left(1\right)+\overset{\infty }{\underset{n=2}{\sum }}\;{\left(1-\delta \right)}^{n-2}n^{2}G\left(n\right)<\infty \text{,} \end{array}$$

where $G\left(n\right)=\underset{i}{sup}\;\sum_{m=1}^{n}g_{i}\left(m\right)$.

So, in this case we have a fast decomposition of the synaptic weights, that is, [27]:

(42) $$\begin{array}{c} \underset{i}{sup}\;\underset{k\geq 1}{\sum }\;\left|V_{i}\left(k\right)\right|\left(\underset{j\notin V_{i}\left(k-1\right)}{\sum }\;\left|W_{j⟶i}\right|\right)<\infty \cdot \end{array}$$

As can be reasonably expected, the results of applying categorization to a data stream are the set of tuples that would result from the union of the individual results that the application would have on the current contents of the stream at any time. Specifically, let *Q* be a categorization query submitted at a time *τ*_*o*_ ∈ *T* to the data stream *S*. Then, the results *Q*^*c*^ to be obtained at time *τ*_*i*_ ∈ *T* are the set of tuples *Q*(*S*(*τ*)) that satisfies the query *Q* from every current content *S(τ)* of the stream until then, that is, [28]:

(43) $$\begin{array}{c} \forall \tau_{i}\in T,Q^{c}\left(S\left(\tau_{i}\right)\right)=\underset{\tau_{0}\leq \tau \leq \tau_{i}}{⋃}\;Q\left(S\left(\tau \right)\right)\cdot \end{array}$$

Obviously, the total valuation for all successive time points is practically unprofitable. So, a strategy is needed that allows for periodic checking of the data so that the answers are calculated periodically. Since all tuples are marked with distinct time milestones, it is possible to evaluate *Q* with a time step ∆_*τ*_. In the k-th iteration, only the intermediate results *Q*^*c*^(*S*(*τ*_*O*_+*k*Δ*τ*)) − *Q*^*c*^(*S*(*τ*_*O*_+(*k* − 1)Δ*τ*)) should be added to the current answer replacing the immediately preceding one, as follows:

(44) $$\begin{array}{c} \Delta Q=\underset{\tau_{0}\leq \tau \leq \tau_{0}+k\Delta \tau }{⋃}\;Q\left(S\left(\tau \right)\right)-\underset{\tau_{0}\leq \tau \leq \tau_{0}+\left(k-1\right)\Delta \tau }{⋃}\;Q\left(S\left(\tau \right)\right)\cdot \end{array}$$

However, the previous formula does not always guarantee correct results. One only must think about what will happen if, over time, newer answers cancel out earlier ones. For example, we consider that all vibrations whose value variation has never exceeded the general threshold index can be requested in the anomaly detection application. But as the data changes dynamically, some tuples included in previous answers may no longer meet the criterion. However, with periodic computation, such results will be retained in all subsequent responses, even though they should typically be discarded.

The following Figure 2 depicts an example of time windows of vibration analysis.

An important innovation in implementing the proposed algorithm is the extension of the GLSM probabilistic algorithm, with the introduction of time intervals and confidence points in the cases where we have samples of independent and identically distributed variables and correspondingly when we have a Markov chain [29]. This extension leads to a system that can extract probabilistic recognition of complex events over time from a stream of low-level events. Accordingly, by introducing time windows and working memory, we modified the existing GLSM approach, where we consider a new class of non-Markovian processes with a countable number of interacting elements, in which and for each time unit, each element can take two values (normal or abnormal), indicating the anomaly state at the given time.

So, the system expands in a nontrivial way for interacting systems, mainly Markovian, and for stochastic chains with variable-length memory that have a finite state space. These features make the proposed GLSM suitable for describing and modeling the temporal evolution of systems, such as tracking anomalies originating from vibration or vibration analysis systems and their intrinsic mapping from biological patterns of neural systems, using a probabilistic tool in a random environment or spacetime.

The application above is founded on the premise that a snapshot of activity, for example, determined by a snapshot of vibrations, might lead to incorrect identification owing to sensor unreliability or inaccuracy, as well as a variety of extraneous events that can generate noise in the data. In terms of the monitoring and control of the recognition process, such occurrences of misidentification of activities might result in unwarranted delays and slow operations. Therefore, there is a need for a more robust identification that identifies the time intervals within which a high-level activity takes place. As a result, we provide a probabilistic technique for computing events based on time intervals.

Specifically, the probability of an interval *I*_*LTA*_=[*i*, *j*] of an LTA activity with length(*I*_*LTA*_)=*j* − *i*+1 time instants is defined as [30]:

(45) $$\begin{array}{c} P\left(I_{LTA}\right)=\frac{\overset{j}{\underset{k=i}{\sum }}\;P\left(holdsAt\left(LTA,k\right)\right)}{\;length\left(I_{LTA}\right)}\cdot \end{array}$$

In other words, the probability of an interval equals the average of the probabilities of each instant in time it contains. More generally, a maximum likelihood interval *I*_*LTA*_=[*i*, *j*] of an LTA activity is an interval such that, given a probability threshold *𝒯* ∈ [0,1], *P*(*I*_*LTA*_) ≥ *𝒯* and there is no other interval *I*_*LTA*_′ such so that *P*(*I*_*LTA*_′) ≥ *𝒯* and *I*_*LTA*_is a subinterval of *I*_*LTA*_′.

A consequence of the maximum likelihood interval criterion above is that such intervals can overlap. So, we keep only one from each set of overlapping intervals, using interval reliability as a selection criterion. The reliability of an interval is defined as the product of its length times its probability [31]:

(46) $$\begin{array}{c} Cred\left(I_{LTA}\right)=length\left(I_{LTA}\right)\cdot P\left(I_{LTA}\right)=\underset{k}{\sum }\;P\left(holdsAt\left(LTA,k\right)\right)\text{,} \end{array}$$

where *k* are the time instants of the interval *I*_*LTA*_. Therefore, for each set of overlapping maximum likelihood intervals *S*={*I*_1_, *I*_2_,…, *I*_*k*_}, we choose the one with the largest confidence value, or briefly the interval *I*_*LTA*_ with confidence $Cre\;d\;\left(I_{LTA}\right)=\max_{i}\left(Cre\;d\left(I_{i}\right)\right)$ for each *i*=1,…, *k*.

It should be noted that when the interactions between the systems are represented by a critically directed random graph with a large but finite number of components, the proposed framework yields an explicit upper bound for the correlation between successive intervals between spikes that is consistent with previous empirical findings of the process.

Applying the Monte Carlo algorithm [32], we obtain the bootstrap estimator of the standard deviation:

(47) $$\begin{array}{c} {\hat{\sigma }}_{B}={\left(\frac{\overset{B}{\underset{b=1}{\sum }}\;{\left\{{\hat{\theta }}^{*}\left(b\right)-{\hat{\theta }}^{*}\left(\cdot \right)\right\}}^{2}}{B-1}\right)}^{1/2}\text{,} \end{array}$$

where:

(48) $$\begin{array}{c} {\hat{\theta }}^{*}\left(\cdot \right)=\frac{\overset{B}{\underset{b=1}{\sum }}\;{\hat{\theta }}^{*}\left(b\right)}{B}\cdot \end{array}$$

After calculating the estimators using bootstrap, we may construct confidence intervals as follows [33]:

(49) $$\begin{array}{c} \theta \in \left[{\hat{G}}^{-1}\left(\frac{\alpha }{2}\right),{\hat{G}}^{-1}\left(1-\frac{\alpha }{2}\right)\right]\text{,} \end{array}$$

as an approximate 1 − *α* central interval for *θ*. This is the percentile method. Let $\hat{G}\left(s\right)$ be the parametric bootstrap cumulative distribution function of ${\hat{\theta }}^{*}\text{:}$

(50) $$\begin{array}{c} \hat{G}\left(s\right)={Prob}_{*}\;\left\{{\hat{\theta }}^{*}<s\right\}\text{,} \end{array}$$

where Prob_*∗*_ denotes the probability calculated according to the bootstrap distribution of ${\hat{\theta }}^{*}$.

We assume that for every integer n⩾1, the weights *W*_*n*_ are interchangeable. Based on the vector of weights *W*_*n*_, the generalized bootstrap mean corresponding to this vector will be the following:

(51) $$\begin{array}{c} {\bar{X}}_{W,n}=\frac{1}{n}\overset{n}{\underset{i=1}{\sum }}\;W_{n,i}X_{i}\cdot \end{array}$$

So, the weights *W*_*n*_ will satisfy the following conditions:

(52) $$\begin{array}{c} \left(W_{I}\right)W_{n,i}⩾0,i=1,2,\ldots ,n,n⩾1\text{,}\\ \left(W_{II}\right)\;\overset{n}{\underset{i=1}{\sum }}\;W_{n,i}=n\text{,}\\ \left(W_{III}\right)\;\frac{1}{n}\overset{n}{\underset{i=1}{\sum }}\;{\left(W_{n,i}-1\right)}^{2}{⟶}_{P}c^{2}\;as\;n⟶\infty \cdot \end{array}$$

It should be said that the bootstrap method with a weighted Poisson distribution was used in the proposed application carried out in the context of this work.

The proposed GLSM is implemented in a deep neural architecture with fully connected layers that unfold in time. The sending of information is carried out based on the generation of an action potential in the body of the presynaptic cell. Whenever a spike propagates through the axon, the firing of the neurons causes a series of actions in the postsynaptic cell, while the membrane rapidly equalizes the postsynaptic potential, at which point the membrane is depolarized. Changes in synaptic plasticity are associated with various forms of memory, as well as short or long memory, flash memory, etc.

Training is performed based on the general backpropagation through time (BPTT) approach so that the neural network stabilizes in time by stacking identical copies of trained neurons. In particular, the matrices of the system weights *w*_*ij*_^in^, *w*_*ij*_, *w*_*ij*_^out^, *w*_*ij*_^back^ remain the same in all copies of the layers. The training data consists of a time series of input-output samples that take the following form:

(53) $$\begin{array}{c} u\left(n\right)={\left(u_{1}\left(n\right),\ldots ,u_{K}\left(n\right)\right)}^{\prime },d\left(n\right)\\ {=\left(d_{1}\left(n\right),\ldots ,d_{L}\left(n\right)\right)}^{\prime }n=1,\ldots ,T\cdot \end{array}$$

The training process starts from the first level and continues gradually to the next levels of the stack that have been acquired by the unfolding of the levels over time. In each copy of the layers at time *n*, the input *u*(*n*) is introduced, the *x*(*n*) of the intermediate layers is calculated based on *u*(*n*), *x*(*n* − 1) and *y*(*n* − 1) and finally, the output *y*(*n*) is calculated. The error function that is being reduced is as follows:

(54) $$\begin{array}{c} E=\underset{n=1,\ldots ,T}{\sum }\;{\left\|d\left(n\right)-y\left(n\right)\right\|}^{2}=\underset{n=1,\ldots ,T}{\sum }\;E\left(n\right)\text{,} \end{array}$$

but the meaning of *t* has changed from the training instance to time. For each activation of nodes *x*(*n*), *y*(*n*), the error propagation is given by the following formulas. For the input nodes in the time plane T:

(55) $$\begin{array}{c} \delta_{j}\left(T\right)={\left.\left(d_{j}\left(T\right)-y_{j}\left(T\right)\right)\frac{\partial f\left(u\right)}{\partial u}\right|}_{u=z_{j}}\left(T\right)\cdot \end{array}$$

For the output nodes in time plane *T*:

(56) $$\begin{array}{c} \delta_{i}\left(T\right)={\left.\left[\overset{L}{\underset{j=1}{\sum }}\;\delta_{j}\left(T\right)w_{ji}^{out\;}\right]\frac{\partial f\left(u\right)}{\partial u}\right|}_{u=\lambda_{i}\left(n\right)}\text{,} \end{array}$$

For the internal nodes in the time plane *T*:

(57) $$\begin{array}{c} \delta_{j}\left(n\right)={\left.\left[\left(d_{j}\left(n\right)-y_{j}\left(n\right)\right)+\overset{N}{\underset{i=1}{\sum }}\;\delta_{i}\left(n+1\right)w_{ij}^{back}\right]\frac{\partial f\left(u\right)}{\partial u}\right|}_{u=z_{j}\left(n\right)}\text{,} \end{array}$$

for the output nodes of previous time levels:

The maximum value that the current nodes can reach can be realized based on the following settings:

(58) $$\begin{array}{c} w_{ij}=w_{ij}+\gamma \overset{T}{\underset{n=1}{\sum }}\;\delta_{i}\left(n\right)x_{j}\left(n-1\right)\text{,}\\ w_{ij}^{in}=w_{ij}^{in}+\gamma \overset{T}{\underset{n=1}{\sum }}\;\delta_{i}\left(n\right)u_{j}\left(n\right)\text{,}\\ \begin{array}{c} w_{ij}^{out\;}=w_{ij}^{out\;}+\gamma \times \left\{\begin{array}{c} \overset{T}{\underset{n=1}{\sum }}\;\delta_{i}\left(n\right)u_{j}\left(n\right),\\ \overset{T}{\underset{n=1}{\sum }}\;\delta_{i}\left(n\right)x_{j}\left(n-1\right), \end{array}\right.\\ w_{ij}^{back}=w_{ij}^{back}+\gamma \overset{T}{\underset{n=1}{\sum }}\;\delta_{i}\left(n\right)y_{j}\left(n-1\right)\cdot \end{array} \end{array}$$

Figure 3 shows the result of the process after using the proposed algorithm in modeling the problem of discovering anomalies in vibration data.

To compare the method with competitors and to confirm its superiority, the comparison Table 1 is shown below.

In conclusion, and as can be seen from the results and analyses presented above, the proposed model, considering the objective difficulties raised in this research, is a significant and powerful anomaly recognition model capable of coping with complex situations. It is essential to state that the repeated execution of these training epochs results in a complex nonlinear dynamic system that can often deviate from the desired behavior. Therefore, bifurcations are likely to form when the initialization values of the network weights are quite different from the dynamics of the system we aim to model. Near such bifurcations, gradient information can become essentially useless, dramatically reducing convergence. The fault may develop suddenly near such critical points because of the crossing boundaries of the branches. Nevertheless, modeling with spiking neural networks where idealized neurons interact with sporadic near-instantaneous discrete events in confidence intervals is guaranteed to converge to a minimum local error. This observation cannot occur with feedforward networks because they model only simple functions and not dynamical systems.

## 5. Conclusion

In this paper, we examine threats to the digital security of petroleum infrastructure protection services. Specifically, we presented a deep spiking neural network anomaly detection method by simulating the human brain and the way neural information is processed and transmitted. We utilized a particularly innovative form of the Galves–Löcherbach Spiking Model (GLSM), which is a spiking neural network model with intrinsic stochasticity, ideal for modeling complex spatiotemporal situations.

The proposed model is a significant and powerful anomaly recognition model capable of coping with complex situations, despite the objective difficulties raised in this research. The repeated execution of these training epochs leads in a complicated nonlinear dynamic system that frequently deviates from the planned behavior. Therefore, bifurcations are likely to occur when the initialization values of the network weights are significantly dissimilar to the dynamics of the system we are attempting to mimic. Near to such bifurcations, gradient information may become essentially meaningless, hence drastically lowering convergence. Due to the crossing borders of the branches, the fault may form suddenly close to such crucial spots. However, modeling with spiking neural networks in which idealized neurons interact with random near-instantaneous discrete events in confidence intervals is guaranteed to converge to a minimum local error.

Conventional deep learning relies on stochastic gradient descent and error backpropagation, which requires differentiable activation functions. Consequently, modifications are required to reduce activations to binary values. Integrating the timing of asynchronous operations into the training process is only performed by asynchronous spiking neural networks. Such networks share the discontinuous nature of data but not the asynchronous operation mode of spiking neural networks. In contrast to deterministic models for spiking neural networks, a probabilistic model defines the outputs of all spiking neurons as jointly distributed binary random processes. The joint distribution is differentiable in the synaptic weights, and, as a result, so are principled learning criteria from statistics and information theory, such as likelihood function and mutual information. The change in weight distribution during the learning process is based on the weight distribution of each time interval. The maximization of such measures can apply to arbitrary topologies and does not require the implementation of backpropagation mechanisms. Hence, a stochastic viewpoint has significant analytic advantages, which translate into deriving flexible learning rules from first principles. These rules recover as exceptional cases in the theoretical neuroscience literature of the proposed model.

On the other hand, a learning rule is a local binary random process whose operation can be decomposed into atomic steps carried out in parallel at distributed processors based only on locally available information and limited communication on the connectivity graph. Local knowledge at a neuron includes the membrane potential, the feedforward filtered traces for the incoming synapses, the local feedback filtered trace, and the local model parameters. Besides local signals, learning rules may also require global feedback signals. Finally, the proposed model can use an iteration rule for a rate-coded error signal on a more extended “macro” time scale and combines this with an update on a shorter “micro” time scale which captures individual spike effects.

As an extension of the envisioned system in the future, future study should include further modification of the GLSM parameters to develop a categorization process that is even more effective and rapid [34]. For the suggested framework to fully automate the process of locating APT attacks, it must also be expanded based on methodologies for selfimprovement and parameter redefinition. In the direction of future expansion, the creation of an additional cross-sectional anomaly analysis system is a further feature that may be examined. This could act diametrically opposed to the GLSM classifier's ideology and increase the system's effectiveness.

## Figures and Tables

**Figure 1:** Vibration data.

**Figure 2:** Time windows of vibration analysis.

**Figure 3:** Anomalies plot.

**Table 1:** Anomalies detection performance metrics.

Classifier	Accuracy (%)	RMSE	Precision	Recall	F-score	AUC
GLSM	97.88	0.0710	0.987	0.987	0.987	0.9883
Autoencoder	95.92	0.0847	0.960	0.960	0.960	0.9798
LSTM	95.08	0.0891	0.951	0.951	0.952	0.9732
CNN	94.59	0.0928	0.946	0.946	0.947	0.9781
One class SVM	93.26	0.0933	0.933	0.934	0.933	0.9590
Isolation forest	92.51	0.0925	0.925	0.925	0.925	0.9519

## Data Availability

The data used in the proposed approach are available from the corresponding author upon reasonable request.
